# Effect of carbon-enriched digestate on the microbial soil activity

This article has been retracted.

**DOI:** 10.1371/journal.pone.0252262

**Published:** 2021-07-02

**Authors:** Jiri Holatko, Tereza Hammerschmiedt, Antonin Kintl, Subhan Danish, Petr Skarpa, Oldrich Latal, Tivadar Baltazar, Shah Fahad, Hanife Akça, Suleyman Taban, Eliska Kobzova, Rahul Datta, Ondrej Malicek, Ghulam Sabir Hussain, Martin Brtnicky

**Affiliations:** 1 Department of Agrochemistry, Soil Science, Microbiology and Plant Nutrition, Faculty of AgriSciences, Mendel University in Brno, Brno, Czech Republic; 2 Department of Geology and Soil Science, Faculty of Forestry and Wood Technology, Mendel University in Brno, Brno, Czech Republic; 3 Agricultural Research, Ltd., Troubsko, Czech Republic; 4 Department of Soil Science, Faculty of Agricultural Sciences and Technology, Bahauddin Zakariya University, Multan, Punjab, Pakistan; 5 Hainan Key Laboratory for Sustainable Utilization of Tropical Bioresource, College of Tropical Crops, Hainan University, Haikou, China; 6 Department of Agronomy, the University of Haripur, Khyber Pakhtunkhwa, Pakistan; 7 Department of Soil Science and Plant Nutrition, Faculty of Agriculture, Ankara University, Ankara, Turkey; 8 Department of Agronomy, Faculty of Agricultural Sciences and Technology, Bahauddin Zakariya University Multan, Punjab, Pakistan; 9 Institute of Chemistry and Technology of Environmental Protection, Faculty of Chemistry, Brno University of Technology, Brno, Czech Republic; Government College University Faisalabad, Pakistan, PAKISTAN

## Abstract

**Objectives:**

As a liquid organic fertilizer used in agriculture, digestate is rich in many nutrients (i.e. nitrogen, phosphorus, sulfur, calcium, potassium); their utilization may be however less efficient in soils poor in organic carbon (due to low carbon:nitrogen ratio). In order to solve the disadvantages, digestate enrichment with carbon-rich amendments biochar or humic acids (Humac) was tested.

**Methods:**

Soil variants amended with enriched digestate: digestate + biochar, digestate + Humac, and digestate + combined biochar and humic acids—were compared to control with untreated digestate in their effect on total soil carbon and nitrogen, microbial biomass carbon, soil respiration and soil enzymatic activities in a pot experiment. Yield of the test crop lettuce was also determined for all variants.

**Results:**

Soil respiration was the most significantly increased property, positively affected by digestate + Humac. Both digestate + biochar and digestate + Humac significantly increased microbial biomass carbon. Significant negative effect of digestate + biochar (compared to the control digestate) on particular enzyme activities was alleviated by the addition of humic acids. No significant differences among the tested variants were found in the above-ground and root plant biomass.

**Conclusions:**

The tested organic supplements improved the digestate effect on some determined soil properties. We deduced from the results (carbon:nitrogen ratio, microbial biomass and activity) that the assimilation of nutrients by plants increased; however, the most desired positive effect on the yield of crop biomass was not demonstrated. We assume that the digestate enrichment with organic amendments may be more beneficial in a long time-scaled trial.

## 1. Introduction

Digestate is a residual waste material from anaerobic biogas production, used as a fertilizer rich in nitrogen (N) compounds (inorganic N is mostly in the form of ammonia), phosphorus (P, available to plants is increased during anaerobic digestion) sulfur (S), calcium (Ca), potassium (K), magnesium (Mg) and microelements [1]. The use of digestate in agriculture has a positive effect on the growth and production of crops [2]. The application of digestate to soil showed also other beneficial effects: reduction of bulk density, increase in hydraulic conductivity, water retention capacity [3] and stability of aggregates [4]. Digestate may increase the content of organic matter (humus) [4] and support microbial activities in the soil comparably to livestock fertilizers (pig manure, cow manure) [5].

However, the digestate carbon (C) content may decrease during anaerobic digestion and cause a reduced input of organic C into the soil in comparison to fertilization with manures or compared to direct incorporation of undigested crop residues [6]. C-rich organic amendments (e.g. biochar) with a potential to sequester C [7] could be applied together with digestate and compensate this disadvantage by higher stabilization of both C [8] and N [9]. It was reported that amendment of digestate and biochar increased both total organic carbon (TOC) and soil C turnover in comparison to the sole digestate application [10]. Nevertheless, other authors referred about the reduction of soluble compounds (dissolved organic C and phenols) due to the addition of biochar to digestate. This reduced biomass and activity of the soil microbiota [11] or sloweddown mineralization and release of biochar-adsorbed nutrients in the short-term application [12]. These temporary effects of digestate and biochar co-application to soil lead to a slightly lower yield [12], above-ground biomass (AGB) and total N off-take [13]. Nevertheless, the long effect of biochar on digestate could result in a higher soil C sink by increasing the TOC content [11]. It could bring the benefit in sustaining soil fertility, high soil organic matter (SOM) and gradually releasing micronutrients [12].

Therefore, this research aimed to evaluate the effect of digestate pre-treated (before application) with biochar on the soil properties and plant growth. Moreover, digestate was reported to form smaller amounts of humic acids (HA) with the lower C:N ratio compared with the composted organic materials [14]. Amending arable soil with biochar or digestate results in chemical and structural changes of humic substances [15] and increased levels of humic and fulvic acids and soil TOC [16]. In saline soils, digestate combined with Ca humate followed by humic acid treatments showed greater microbial biomass carbon (MBC), microbial biomass nitrogen (MBN), soil enzyme activities [17]. Thus, we found interesting to increase the C content of digestate by adding exogenous HA with a high C:N ratio, primarily because we observed that the negative priming effect of high biochar dose on C mineralization in the soil was alleviated by the simultaneous addition of HA [18]. Therefore, similarly to biochar active as a sorbent and C-rich soil organic amendment, the humic acid-based material was used to modify fertilizing and biological properties of digestate. We also tested the impact of the combined biochar and HA-enrichment of digestate on the excessive C stabilization and retarded mineralization, under the conditions of the short-term pot experiment. Thus, the final objectives were as follows: (1) to compare the effect of untreated control digestate and digestate mixed with either biochar, HA or both organic matters on soil properties; and (2) to evaluate the presumed beneficial effect of mixed digestates on the soil nutrient content and on the crop yield.

## 2. Material and methods

### 2.1 Soil amendments

The following amendments were used in this study to modify the digestate and to be co-applied with it into the soil: biochar pyrolyzed at a moderate temperature (approx. 600–650°C), from agricultural grain waste (Sonnenerde GmbH, Austria); HA-based product Humac AGRO (mined commercial stimulator of soil fertility, prepared from leonardite-oxihumolite—Envi Produkt Ltd., Czech Republic) [18]; and digestate (produced from gastro-waste) from the continuous mesophilic (~ 40°C) biogas plant (Czech Republic). The amendments were treated according to the procedure described in Chapter 2.2. The field soil was collected near the town Troubsko, Czech Republic (49°10’28"N 16°29’32"E), on private land in autumn 2018. We confirm that the owner of the land gave permission to collect the soil.

### 2.2 Digestate preparation

The enriched digestate variants were prepared by post-fermentation incubation of the basic digestate. The incubation took place in tightly closeable vessels (volume of 50 dm^3^) which were filled (according to experimental variants) with: (I) 10 dm^3^ of (control) digestate; (II) 10 dm^3^ of digestate + 4 kg of biochar; (III) 10 dm^3^ of digestate + 4 kg of biochar + 100 g of Humac; (IV) 10 dm^3^ of digestate + 100 g of Humac. The digestate was thoroughly mixed with the organic amendmend(s), the vessels were sealed and left at 17.4–20.2° C for 6 weeks. All variants were performed in triplicates, their properties were determined at the beginning of the experiment and are shown in Table 1.

**Table 1:** Properties of digestates used in the pot experiment.

component/unit	(I) control digestate	(II) digestate + biochar	(III) digestate + biochar + Humac	(IV) digestate + Humac
dry matter [%]	6.0	15.0	15.8	6.8
TN [g·kg^-1^]	6.5	6.8	7.6	5.0
N_norg_ [g·kg^-1^]	0.74	0.65	0.48	0.98
N-NO_3_ [g·kg^-1^]	0.22	0.25	0.06	0.37
N-NH_4_ [g·kg^-1^]	0.52	0.40	0.42	0.61
P [g·kg^-1^]	12.8	13.9	7.9	14.0
S [g·kg^-1^]	14.3	15.1	17.5	16.2
Ca [g·kg^-1^]	19.2	21.1	11.5	24.1
Mg [g·kg^-1^]	1.55	1.50	1.63	2.13
Na [g·kg^-1^]	5.99	6.10	1.15	6.00
K [g·kg^-1^]	22.6	24.2	6.8	26.6

### 2.3 Soil substrate preparation

The growth substrate used for this pot experiment consisted of topsoil (0–15 cm) mixed with quartz sand. The field soil was collected near the town Troubsko, Czech Republic (49°10’28"N 16°29’32"E). The soil type was clayey to loamy, modal brown earth. In order to remove coarse particles, the soil was sieved through a grid sized 2.0 mm. The sieved soil was mixed with the fine quartz sand (0.1–1.0 mm) (1:1, w/w) to increase nutrients content and enhance the effect of fertilization. Soil properties determined before the start of the experiment were as follows: soil macronutrients (in g·kg^-1^): TC 7.0, TN 0.80, P 0.049, S 0.073, Ca 1.60, Mg 0.118, K 0.115, Si 220.0; N forms (in mg·kg^-1^)–N_inorg_ 32.8, N-NO_3_ 29.6, N-NH_4_ 3.2; soil reaction = pH (CaCl_2_) 7.3.

### 2.4 Pot experiment preparation

Four different soil variants were prepared for the experiment which was carried out in the pots (volume 1 dm^3^): top diameter 11 cm, bottom diameter 9 cm, height 13 cm [19]. The pots were filled up with 1 kg of the growth substrate (soil-sand mixture), mixed thoroughly with the particular variants of digestates as follows: (1) control digestate 40 ml (per pot; equaled 50 m^3^·ha^-1^) (2) digestate + biochar 40 ml (biochar equaled 20 t·ha^-1^); (3) digestate + biochar + Humac 40 ml (biochar equaled 20 t·ha^-1^; Humac equaled 1 t·ha^-1^); (4) digestate + Humac 40 ml (Humac equaled 1 t·ha^-1^). Each variant was preparedin 3 repetitions (pots).

Each pot was watered with 100 ml of demineralized water. The test crop was lettuce (*Lactuca sativa* L. var. *capitata* L.) cv. Smaragd. 2-day sprouting of lettuce seeds on the wet filter paper preceded their sowing into a depth of approx. 2 mm in each pot. The incubation took place in the growth chamber under the following controlled conditions: full-spectrum stable white LED lighting, intensity 20 000 lx [20], ~ 200 μmol·m^-2^·s^-1^ [21]). Conditions of the environment were: temperature 18/22°C (night/day), relative humidity 70% [22], photoperiod 12 h [23]. Pot placement in the growth chamber was randomized. 10-day-old seedlings were reduced to only one (most robust) per each pot. Each pot was manually wateredwith 50 ml of demineralized water every other day. The pots were variably rotated once per week [24]. 6 weeks after sowing, the plants were harvested [25]. A soil sample was collected from each pot.

### 2.5 Plant biomass

Lettuce shoots were cut at ground level and roots were gently cleaned from the soil and washed with water [24]. The shoots and roots were weighted separately on analytical scales to determine fresh AGB (of lettuce shoots) and fresh root biomass.

### 2.6 Soil sampling and preparation

Soil samples were collected after the harvest of lettuce (1 mixed sample per pot). The samples were homogenized by sieving through a 2 mm mesh under sterile conditions. Samples for enzyme activity assays (β-glucosidase (GLU), urease (Urea), arylsulfatase (ARS), phosphatase (Phos) and N-acetyl-β-D-glucosaminidase (NAG)) were freeze-dried. Samples for the dehydrogenase (DHA) assay, MBC determination and respiration (basal (BR) and substrate-induced (SIR)) measurement had been stored at 4°C for 14 days before they were analyzed.

### 2.7 Chemical, biological, and statistical analyses

Soil properties were determined, and the obtained data statistically analyzed using methods listed in the Table 2, specifications of which were identical to our previously published research [18]. Four to nine replications (values of independent measurements) were used at calculating the Multivariate analysis of variance (MANOVA). The Kolmogorov-Smirnov test was used for testing the Normality, and the Anderson-Darling normality test was used to test homoscedasticity.

**Table 2:** Determined soil properties, methods used for measurement and statistics, relevant references.

Property	Method	Unit	Reference
Total soil carbon	dry combustion using LECO TruSpec analyzer (MI USA)	mg∙g^-1^	ISO 10694: 1995 [26]
Total soil nitrogen			ISO 13878: 1998 [27]
Microbial biomass carbon	fumigation extraction method	mg∙g^-1^	[28]
Basal soil respiration	MicroResp® device	μg CO_2_·g^-1^·h^−1^	Technical Manual v2.1; [29]
Substrate induced soil respiration	MicroResp® device + inducers (sugars, amino acids)		
Soil enzyme activities (GLU, NAG, Phos, ARS, Urea)	Microplate incubation, Vis spectrophotometry	μmol PNP·g^-1^·h^-1^, μmol NH_3_·g^-1^·h^-1^	ISO 20130: 2018 [30]
Soil enzyme activity—DHA	triphenyl tetrazolium chloride (TTC)-based method	μg TPF·g^-1^·h^-1^	[31, 32]
**Processing**	**Tool**	**Method**	**Reference**
Statistical analysis	Program R version 3.6.1.	Multivariate analysis of variance (MANOVA), principal component analysis (PCA), one-way analysis of variance (ANOVA), Duncan’s multiple range test, Pearson correlation analysis	[18]

## 3. Results

The results analyzed by MANOVA showed significant differences between the experimental variants in all determined properties except of DHA and fresh plant AGB, root) biomass (S1 Table). The results of Pearson’s correlation analysis are in the (S1 Fig) and mentioned when the value of the correlation coefficient ρ was: 0.5<ρ<0.7 (moderate correlation) and 0.7<ρ<0.9 (high correlation) [33]. The evaluation of the mutual dependence between the properties and their values in the individual compared experimental variants is shown in the Rohlf PCA Biplot (Fig 1).

**Fig 1:** Rohlf PCA biplot of individuals and variable.

### 3.1 Effects of digestate on the soil nutrients, microbial biomass and plant biomass

Variant (3) amended with digestate + biochar + Humac showed a significantly increased total carbon (TC) content as compared to Variant (1) with the control digestate—Fig 2A. Further, TC was found to exhibit a moderately negative correlation with lysine SIR (Lys-SIR, ρ = 0.5) and a highly positive correlation with the C:N ratio (ρ = 0.78). Rohlf PCA Biplot showed an antagonistic relationship to enzyme activities (mainly Urea and DHA) and to the soil respiration (Fig 1). We assume that when added into the soil, digestate enriched with a high dose of biochar increased the content of recalcitrant C and resulted in C stabilization in the soil and the increased C:N ratio. MBC was significantly increased in variants with the biochar-enriched (2) and HA-enriched (4) digestates as compared to the control–Fig 2C. However, the surplus of C in variant (3) digestate + biochar + Humac seemed to reduce the positive effect of organic amendments on the cycling of nutrientsdue to the excessively high C:N ratio which was adverse to soil microbes (Figs 2B and 1C).

**Fig 2:** **a-f** Total soil carbon **(a)** and nitrogen **(b)**, C:N ratio **(c)**, microbial biomass carbon **(d)**, fresh above-ground **(b)** and root biomass **(f)** mean values with a confidence interval of 95% (error bars). Different letters indicate statistically significant differences in MANOVA at p ≤ 0.05.

Contrarily to TC, total soil nitrogen (TN) content was the highest in the control variant (1), significantly exceeding the values in Variants (2) and (3), where biochar was added (Fig 2B). TN exhibited a moderately negative correlation with MBC (ρ = -0.62) and a moderately positive correlation with ARS (ρ = 0.5) and Phos (ρ = 0.55). Rohlf PCA Biplot showed an antagonistic relationship to other enzyme activities, to the fresh root biomass and fresh AGB—Fig 1. The biochar-enriched digestates (2) and (3) tended to increase the C:N ratio (Fig 2C). However, the HA-enriched digestate did not increase the C:N in the soil just negligibly, thus leading to just non-significantly decreased TN (Fig 2B) and lower values of MBC (compared to the digestate + biochar variants)–Fig 2D. A positive relationship between TN and enzyme activities was observed, which was contradictory to MBC (Figs 2A, 2D and 4). Less nutrients likely remained available to plants in the control variant, this causing (non-significantly) lower fresh AGB and root biomass (Fig 2E and 2F), which was apparent from the antagonism of biomass and TN in the PCA Biplot analysis (Fig 1). The significantly lowest TN in Variant (3) digestate + biochar + Humac anticipated the highest acquisition of nutrients from the treated soil by plants as the C:N value (13.1) was closest to the soil optimum for plant growth [34]. Therefore, the non-significantly highest fresh AGB and significantly highest root biomass (as compared to the control) was detected in this variant (3) digestate + biochar + Humac (Fig 2E and 2F).

### 3.2 Effects of digestate on the soil microbial activity

BR was significantly increased only in Variant (4) amended with digestate enriched with HA (Fig 3A), as compared to the control. This finding corroborated the presumed negative relationship between plant growth and microbial decomposition. A further evidence was the antagonism between BR and both TC and TN, apparent from Rohlf PCA Biplot (Fig 1). An increased competition for available nutrients may be assumed from the moderately positive correlation between BR and root biomass (ρ = 0.57), which may reflect an induced enlargement of the plant root system. A positive high correlation between BR and all SIRs except of glucose (Glc) and alanine (Ala), was further observed: trehalose SIR (Tre-SIR, ρ = 0.71), N-acetyl-β-D-glucosamine SIR (NAG-SIR,ρ = 0.8), Lys-SIR (ρ = 0.71), and arginine SIR (Arg-SIR, ρ = 0.83). These results showed that all SIRs were again significantly increased (in comparison to the control) only in Variant (4) amended with digestate + Humac (Fig 3B–3E), except of Arg-SIR. Arg-SIR was increased also in Variant (3) amended with digestate + biochar + Humac (Fig 3F). Rohlf PCA Biplot revealed a high antagonism among all determined types of soil respiration (Fig 1).

**Fig 3:** **a-g** Basal **(a)** and substrate-induced respiration: D-glucose **(b),** D-trehalose **(c)**, N-acetyl-β-D-glucosamine **(d),** L-alanine **(e),** L-lysine **(f),** L-arginine **(g)**–M with CI 95% (error bars). Different letters indicate statistically significant differences in MANOVA at p ≤ 0.05.

Soil enzyme activities manifested a narrow positive relationship between one another too, except of urease (Fig 1). There was no significant difference among all variants in the DHA activity (Fig 4A); however, DHA showed a moderately positive correlation with Phos (ρ = 0.53). Which was the only enzyme which exhibited significant differences among all variants, showing the highest activity in the control, descending values from Variant (4) digestate + Humac to Variant (3) digestate + biochar + Humac and the lowest values in Variant (2) digestate + biochar (Fig 4F). Phos correlated moderately positively with ARS (ρ = 0.66), NAG (ρ = 0.69), and GLU (ρ = 0.66), and moderately negatively with C:N (ρ = - 0.59). The positive relationship to TN was already mentioned and the Phos values responded to the TN content in the soil of all variants. From other 4 enzymes which showed antagonism to the C:N ratio on Rohlf PCA Biplot (Fig 1), only NAG exhibited a moderately negative correlation with C:N (ρ = - 0.5). These enzymes showed either lower activity (as compared to the control) in all variants amended with the enriched digestate (ARS, NAG) or only in Variant (2) digestate + biochar (Urea)–Fig 4B–4D. We deduced that the highest TC was accompanied by the lowest enzyme activities (significant for ARS, Urea) involved in the decomposition of nutrient sources (S, N) other than carbon. Nevertheless, GLU was more active in the presence of humic acids (in comparison to the control and the digestate + biochar variant), however it was non-significant (Fig 4E). The carbon sequestration was presumably achieved by biochar-induced stabilization of soil SOM and hindrance from the microbial decomposition.

**Fig 4:** **a-f** Enzyme activities of: dehydrogenase **(a)**, arylsulfatase **(b),** urease **(c)**, N-acetyl-β-D-glucosaminidase **(d),** β-glucosidase **(e),** phosphatase **(f)**–M with CI 95% (error bars). Different letters indicate statistically significant differences in MANOVA at p ≤ 0.05.

## 4. Discussion

Some studies reported increased crop yield due to the application of digestate with C-rich organic (i.e. biochar) amendment [12, 35]. Our results indicate this trend as well; however, no significant difference was observed. In this experiment, we evidenced that the access of C from biochar- and mainly from biochar + Humac-enriched digestate lead to putative initial increase in the microbial abundance and biomass (Fig 2), which was further accompanied with the decreased enzyme (Phos, Urea, ARS, NAG) and respiratory activity of soil microorganisms (Figs 2 and 3). The reduced CO_2_ emission after the application of biochar amended with N-rich organic matter into the soil was already reported [36]. Presumably the labile and available C from biochar, digestate or HA was utilized by the soil microflora and further decomposition was abolished due to the recalcitrance and enzyme-inhibiting effect of biochar material, as it was referred [37]. Only the access of HA-derived C preserved the non-decreased C decomposing activity of GLU even in the presence of biochar (Fig 3E). The sole HA-enrichment of digestate resulted in amended soil in a significantly higher microbial respiratory activity (Fig 3). Some authors [38, 39] referred on a similar positive effect of HA-rich amendment on the soil respiration and microbial carbon under access of N and P which were also abundant in the digestate in our experiment.

Nevertheless, we assumed that the inhibited microbial decomposition of SOM, indicated by the reduced enzyme activity (Fig 4) and respiratory potential, was accompanied by the decreased nitrification and acquisition of N from digestate by the soil microflora, as it was reported in earlier studies [40]. The preservation of available N presumably allowed higher assimilation by plants. This assumption can be deduced from the higher C:N in biochar-amended variants (2, 3), which is known to be less desirable for microbial nutrition but beneficial for plant nutrition. There is a study which reported on the decreased cumulative N mineralization rate in the digestate-amended soil with a high C:N ratio [41]. Our observations agreed with the reported short-acting N-fertilizing effect of digestate, which resembles fertilizing features of urea [41]. Although the biochar-enriched digestates decreased TN (Fig 2B), they had a potential to stabilize and sequester nutrients including N-ammonium (N-NH_4_), a prevalent form of plant-available N in digestate, in the same way as it was reported [42, 43]. Such effect on N-NH_4_retention might be enhanced by the HA amendment and we presumed retardation of N-NH_4_oxidation in digestate, similar to that reported for urea (amendment) [44, 45]. We documented this with values of fresh plant (AGB, root) biomass in the digestate + biochar and digestate + biochar + Humac variants which exhibited concurrently the highest C:N ratio. We found a consent with studies referring on partially improved properties of biochar due to digestate co-treatment [46], including improved availability of nutrients [47]. However, not even these studies demonstrated that the higher access to nutrients might lead to the increased crop yield [46–50].

## 5. Conclusions

A significant effect on the BR and the most of SIRs were detected for the digestate variant mixed with HA, the application of which increased the control values in the range from +17% to +173% (average values). The variant of digestate + biochar + Humac showed significantly increased Arg-SIR. Both variants of digestate + biochar and digestate + Humac increased MBC (compared to the control digestate) by +37% and +30%, respectively. A significant increase in TC (compared to the control) was observed only in variant digestate + biochar + Humac.

However, a significant decrease in the soil enzyme activities–ARS, Phos, NAG–was detected in all 3 enriched digestate variants as compared to the control. This decrease did not occur (or was alleviated) in the case of GLU and Urea in the both variants amended with HA. The fresh root and AGB plant biomass did not show any significant change related to the different digestate variants applied; nevertheless, the highest crop yield of digestate + biochar + Humac increased as compared to the control (fresh AGB +24%) and (fresh root biomass +29%). The significantly decreased TN (compared to the control) in the variants with a higher crop yield (digestate + biochar and digestate + biochar + Humac) may indicate increased N assimilation by the plant.

The application of digestate enriched with the organic amendments positively affects soil microbial respiration and abundance. Although the beneficial effect on the crop growth and yield was non-significant, the promising impact of organic supplements on the digestate quality is anticipated and should be further investigated.

## Supporting information

S1 Fig Correlation matrix of soil properties (numbers indicate the Pearson’s correlation coefficient ρ). (TIF)

S1 Table Detailed results after the multivariate analysis of variance MANOVA (ANOVA separately). (XLSX)

## Abbreviations

AGB: above-ground biomass
N-NH_4_: ammonium
N_inorg_: inorganic nitrogen
ARS: arylsulfatase
BR: basal respiration
GLU: β-glucosidase
Ca: calcium
C: carbon
Glc: D-glucose
Tre: D-trehalose
DHA: dehydrogenase
HA: humic acids
Ala: L-alanine
Arg: L-arginine
Lys: L-lysine
Mg: magnesium
M: mean value
MBC: microbial biomass carbon
NAG: N-acetyl-β-D-glucosaminidase
N-NO_3_: nitrate
N: nitrogen
ρ: Pearson’s correlation coefficient
Phos: phosphatase
P: phosphorus
K: potassium
Si: silicon
SOM: soil organic matter
CI 95%: confidence interval 95%
SIR: substrate induced respiration
S: sulfur
TOC: total organic carbon
TC: total carbon
TN: total soil nitrogen
Urea: urease
